# Protocatechuic acid attenuates cerebral aneurysm formation and progression by inhibiting TNF-alpha/Nrf-2/NF-kB-mediated inflammatory mechanisms in experimental rats

**DOI:** 10.1515/biol-2021-0012

**Published:** 2021-02-16

**Authors:** Gang Xiao, Mei Zhang, Xing Peng, Guangyuan Jiang

**Affiliations:** Department of Neurosurgery, Chongqing Traditional Chinese Medicine Hospital, No. 6 Panxi 7 Branch Road, Jiangbei District, Chongqing 400021, People’s Republic of China; Department of Dermatology, Daping Hospital, Army Medical University, Chongqing 400042, China

**Keywords:** cerebral aneurysm, protocatechuic acid, macrophages, inflammatory response mechanisms, chemokines, TNF-α signaling, Nrf-2

## Abstract

Our current research aims to examine whether protocatechuic acid (PCA) can be used as a therapeutic agent for the development of cerebral aneurysm (CA) and to elucidate the mechanisms behind this. We assessed the effects of PCA at 50 and 100 mg/kg on the activation of signaling pathways for tissue necrosis factor (TNF)-α/nuclear factor (NF)-κB/nuclear factor erythroid 2 (Nrf-2) on progression and development in an elastase-induced CA model, accompanied by a high-salt diet to induce hypertension. The expression of inflammatory cytokines, chemokines, tumor necrosis factor-α, interleukins (IL)-8, IL-17, IL-6, IL-1β, and matrix metalloproteinase (MMP)-2 and MMP-9 was analyzed by ELISA, western blot, and reverse transcriptase quantative polymerase chain reaction. The expression levels of antioxidant enzymes and translocation of Nrf-2 were also determined. The group treated with PCA demonstrated a significant (*P* < 0.05) decrease in the aneurysmal size in rats compared to the CA-induced group. We found that PCA treatment suppressed the invasion of macrophage and activation of TNF-α/NF-κB/Nrf-2 signaling pathways. There was a significant decrease (*P* < 0.05) in pro-inflammatory cytokine and chemokine levels in a dose-dependent manner. We found that PCA treatment exerts protective effects by suppressing the development and progression of CA through the inhibition of inflammatory responses in macrophages via TNF-α/NF-κB/Nrf-2 signaling pathways, thus demonstrating that PCA can act as a treatment for CA.

## 1 Introduction

Cerebral aneurysm (CA) is the most common cerebrovascular disease with pathological dilations of cerebral arteries occurring in more than 5% of the population [1]. CA can appear as unruptured [2] with a symptom of chronic headache [3] and as ruptured forms, giving rise to hypertension causing a condition called subarachnoid hemorrhage (SAH) [4,5]. This leads to morbidity and mortality worldwide. The etiology of CA is unclear, but several factors, such as chronic inflammation, hemodynamic changes with endothelial dysfunction [6], oxidative stress, and apoptosis, may contribute to the development of CA [7,8]. It is hypothesized that release of inflammatory cytokines and free radicals disrupts the endothelial intima of blood vessel, causing extracellular matrix remodeling dysfunction [6,7,8,9].

Several studies highlighted the important role of chronic inflammation in the formation and progression of CA [10,11,12,13,14]. In addition, reactive oxygen species (ROS) can damage vascular endothelium contributing to the formation and rupture of CA [15,16]. It is known that ROS plays a significant role in inflammation and vascular smooth muscle dysfunction involving transcriptional factor, nuclear factor erythroid 2 (Nrf-2), because of its endogenous antioxidant effect. Under inflammatory conditions, Nrf-2 translocates from the cytoplasm into the nucleus. This results in the expression of endogenous anti-inflammatory and antioxidant substances [17]. However, the pathogenesis of Nrf-2 in the formation and progression of CA is unclear.

Inflammatory responses are also influenced by the recruitment of nuclear factor (NF)-kB-mediated macrophages. This induces the expression of inflammation-related genes such as monocyte chemoattractant protein-1 (MCP-1), interleukin (IL)-1β, inducible nitric oxide synthase (iNOS), and matrix metalloproteinases (MMPs) [18]. NF-kB-mediated signaling through iNOS and IL-1β expression induces apoptosis of vascular smooth muscle causing endothelium damage with the disruption of elastic lamina [19]. It also mediates the expression of MMP-2 and MMP-9 causing degradation of collagen leading to vascular wall remodeling [20].

Studies have shown that increased levels of expression of tissue necrosis factor (TNF)-α are implicated in the progression of CA. This can be induced by the injection of elastase into the coronary arteries and the aorta of animal, which results in the fragmentation of lamina [21,22,23,24]. Chronic inflammation mediated by TNF-α causes disruption of vessel walls and deposition of plaques. The secretion of TNF-α by T-cells also stimulates other immune cells to secrete TNF-α [25].

These plaques formed at the intersection of cerebral arteries and their curvatures [26] weaken the endothelium causing migration of leukocytes [27], which causes further injury to the vascular smooth muscle through the expression of MMPs. This disrupts the tight endothelial junctions between the vascular walls of cerebrum [25]. In addition, several other conditions such as hemodynamic stress and increase in blood pressure exacerbate the expression of TNF-α leading to the progression of CA.

However, there currently exist no noninvasive therapies, and hence the need to develop new therapies to address the formation and progression of CA. In a routine drug screen for various diseases, the therapeutic use of phytochemicals is growing in popularity, because they have either no or low side effects. Protocatechuic acid (PCA) is a phenolic acid, commonly present in green tea, is one of the main metabolites of catechins found in humans after ingestion of green tea infusions. Its antioxidant and anti-inflammatory effects have been widely recognized [28,29,30,31]. It was proven to show antihypertensive and antioxidant effects against high-salt induced hypertension [32]. PCA has also been shown to be efficient in treating asthma airway remodeling [33]. Through anti-inflammatory, antioxidant, and antiapoptotic mechanisms, PCA was used in protecting against methotrexate (MTX) induced hepatorenal toxicity [34]. It has also proved its effectiveness in reducing paw edema, cotton pellet-induced granuloma, and index of arthritis in rat models [35]. PCA exhibits an antiapoptotic effect through activation of the c-Jun N-terminal kinase (JNK) pathway causing Nrf-2 to translocate from the cytoplasm into the nucleus, which results in the suppression of ROS generation [36,37]. In addition, PCA has anti-inflammatory effect in lipopolysaccharide (LPS) induced BV2 microglia, acting on the activation of NF-κB and MAPK signaling pathways [38].

In patients previously pretreated with PCA, inflammation was noticeably restrained. Moreover, pretreartment had an inhibitory effect on the production of NO and TNF-α secretion in the macrophages, which was induced by LPS-induced acute inflammation and oxidative stress by inhibiting iNOS/NO and cyclooxygenase-2 (COX-2) expression/PGE2 expression involving the NF-κB and MAPK signaling pathways [39]. PCA also demonstrated a novel anti-cancer activity that involves the downregulation of the RAS/Akt/NF-kB pathway. This works by targeting RhoB activation and reducing MMP-mediated cell involvement in cancer cells [39]. Chen et al. demonstrated that oral administration of 50 mg/kg of PCA in mice reached a plasma peak of 73.6 μM [40]. Another study by Leila Safaeian et al. showed that PCA at 50, 100, and 200 mg/kg has antioxidant and antihypertensive effects against dexamethasone-induced hypertension [41]. In addition, the study by Bhattacharjee et al. [42] reported that the treatment with PCA at 50 and 100 mg/kg, p.o. significantly (*P* < 0.05–0.01) promotes glucose metabolism in the skeletal muscle, controlling glycemic and lipid levels. This also causes a decrease in the secretion of pro-inflammatory cytokines and improved myocardial physiology to near normalcy in type II diabetic rats.

With the aforementioned effects, we investigated the protective effects of PCA in CA-induced rats with stereotaxic administration of elastase in cerebrospinal fluid to histologically imitate human CA, with inhibition of TNF-alpha/Nrf-2/NF-kB-mediated inflammatory mechanisms for the suppression of CA formation and SAH at doses of 50 and 100 mg/kg, respectively.

## 2 Materials and methods

### 2.1 Rat IA model

Wistar rats of either sex weighing between 150 and 170 g were treated. Elastase (CAS Number 39445-21-1) and PCA (CAS Number: 99-50-3) were procured from Sigma Aldrich, China. Rats were initially divided into four groups: vehicle control, CA induced, PCA treated (50 mg/kg, orally), and PCA treated (100 mg/kg, orally), with 16 rats in each group. PCA was administered orally to rats 1 week before the induction of CA and continued until the end of the experiment. All test groups were treated with ketamine (80 mg/kg) for inducing anesthesia. Before subjecting the rats to left internal carotid artery ligation, a single stereotaxic elastase injection was administered into the cerebrospinal fluid in the right basal cistern as previously illustrated [43]. For 16 weeks, body weights and body mass index (BMI) of rats were recorded in all four groups.

To cause hypertension, a high-salt diet (4% NaCl in standard animal chow and allowed to drink water) was implemented continuously for all the groups for 4 weeks [44]. The tail-cuff procedure was used in rats to assess the systolic blood pressure both before and during treatment, and again for the next 4 weeks. After 90 days, a blue dye containing bromophenol was administered into the lungs, the Willis circle, and major branches. The vascular wall thickness was determined, and the degree of aneurysm was calculated. Hematoxylin and eosin (H&E) staining was used to perform degenerative transformation evaluations of vessel endothelium.


**Ethical approval:** The research related to animal use has been complied with all the relevant national regulations and institutional policies for the care and use of animals.

### 2.2 ELISA measurements

The standard ELISA kits (Catalogue number, CA8563518G3; Chongqing Mbio Technology Co., Ltd, Chongqing, China) were used for assessing cytokine levels (IL-1β, IL-2, IL-17, IL-8, IL-6, and TNF-α). Tissue samples were obtained from all groups around the COW tissues to determine the concentrations of specific cytokines, including IL-1β, IL-2, IL-17, IL-8, IL-6, and TNF-α, as per the instructions of the supplier (Wuhan Fine Biotech Co., Ltd, China). Similarly, the values for the parameters MMP-2 and MMP-9 were also obtained using the commercial kits (Chongqing Mbio Technology Co., Ltd, Chongqing, China).

### 2.3 RNA isolation and quantitative real-time polymerase chain reaction (qRT-PCR) analysis

The samples were collected around the COW region from control and experimental rat groups. Total mRNA was extracted using TRIzol® reagent (Sigma Aldrich, China) according to the manufacturer’s instructions and stored at −80°C. The cDNA was synthesized using ABScript II synthesis kit (Sigma Aldrich, China) to conduct the qRT-PCR (Applied Bio-systems Real-Time PCR, Thermo-Fisher Scientific, China) analysis using SYBR® Green (Sigma Aldrich, China). Thirty to forty cycles were used for performing qRT-PCR. The first phase involved denaturation of cDNA at 90°C for 30 s preceded by annealing for 30 s at 50°C; finally, the method was extended for 40 s at 70°C. The ΔCt method was used to measure the expression of transcripts normalizing to the internal control of glyceraldehyde 3-phosphate dehydrogenase (GAPDH). The primers (Eurofins MWG Operon, Bangalore, Karnataka, India) used for quantifying specific genes in this study are listed in Table 1.

**Table 1:** Oligonucleotides used in this study

Gene	Primer	Sequence
TNF-α	5′ forward 3′	CATCCGTTCTCTACCCAGCC
	3′ reverse 5′	AATTCTGAGCCCGGAGTTGG
NF‑κB	5′ forward 3′	ACGATCTGTTTCCCCTCATC
	3′ reverse 5′	TGC TTCTCTCCCCAGGAATA
MMP‑2	5′ forward 3′	CTGATAACCTGGATGCAGTCGT
	3′ reverse 5′	CCAGCCAGTCCGATT TGA
MMP-9	5′ forward 3′	TTCAAGGACGGTCGGTATT
	3′ reverse 5′	CTCGAGCCTAGACCCAACTTA
GAPDH	5′ forward 3′	AAGAAGGTGGTGAAGCAGGC
	3′ reverse 5′	TCCACCACCCTGTTGCTGTA
Nrf-2	5′ forward 3′	CACATCCAGTCAGAAACCAGTGG
	3′ reverse 5′	GGAATGTCTGCGCCAAAAGCTG
INF-γ	5′ forward 3′	GGCAAAAGGACGGTAACACG
	3′ reverse 5′	TCTGTGGGTTGTTCACCTCG
SM22	5′ forward 3′	ATCCTATGGCATGAGCCGTG
	3′ reverse 5′	CAGGCTGTTCACCAACTTGC

### 2.4 Western blotting assay

Protein lysates from the entire COW were obtained, incubated with ice-cold lysis buffer containing 1 mm phenylmethanesulfonyl fluoride (PMSF) and centrifuged at 4°C for 15 min. The protein concentration was determined using Pierce™ BCA Protein Assay kit (CAT No. 23225; Thermo Fisher Scientific, China). Proteins were then separated using a 10% sodium dodecyl sulfate (SDS) - polyacrylamide-based discontinuous gel and western transferred onto 0.3 μm polyvinylidene fluoride or polyvinylidene difluoride (PVDF) membranes. After blocking with 4% (w/v) bovine serum albumin in a mixture of tris-buffered saline and Tween 20 at room temperature, the membranes were incubated overnight at a temperature of 4°C with primary antibodies. After washing, membranes were incubated with horseradish peroxidase-conjugated secondary antibodies at room temperature for 1 h. To visualize proteins, ECL western blotting substrate (BioVision, Inc, Milpitas, CA, USA) was used. The following primary antibodies were used to perform this assay: NF‑κB (#N8523; 1:1,000, Sigma Aldrich, China), β-actin (#SAB3500350; 1:5,000, Sigma Aldrich, China), Lamin B (#SAB5700147; 1:10,000, Sigma Aldrich), MMP-9 (#SAB5700152; 1:2,000, Sigma Aldrich, China), and GAPDH (#AB2302; 1:5,000, Sigma Aldrich, China). To examine the expression of nuclear transcription factor Nrf-2, nuclear and cytoplasmic proteins were isolated separately. Gel electrophoresis was used to differentiate the lysates of cells and then transferred to the PVDF. The membranes were probed with anti-Nrf-2 (#ABE1845; 1:500, Sigma Aldrich, China), anti-NADPH (#ab109225; 1:2,000, ElabScience, Hubei, China), and anti-αSMA antibodies (#ab5694; 1:5,000, ElabScience, Hubei, China). The membranes were visualized with improved chemiluminescence, followed by X-ray film for imaging. The results were analyzed using ImageJ.

### 2.5 H&E and immunohistochemical staining

The extracted tissues were sliced into 5 μM sections and placed on polylysine-coated slides until treatment with H&E. The tissues were then stained with hematoxylin solutions for 7 h at temperatures between 50 and 70°C and then washed with tap water till the water was colorless. Next, 10% acetic acid and 85% ethanol were used for 2 and 10 h for differentiation of the tissue, and tissues were then washed with tap water. We saturated the tissue in the lithium carbonate solution for 10 h and then washed it with tap water. Eventually, staining was done for 48 h with the eosin solution. The tissue slices were dehydrated twice for 30 min with 95% ethanol and then immersed in xylene at 50–70°C for 1 h, accompanied by paraffin for 10 h. The stained tissues were then imaged using microscopy.

Paraffin-embedded sections in Histoclear solution were heated overnight to 50°C and deparaffinized for 5–10 min. The sections were rehydrated using 100% alcohol twice for 10 min, followed by 95%, 90%, 70% of alcohol for 10 min respectively. Subsequently the sections were re-hydrated with water for 5 min. The activity of endogenous peroxidase was inactivated by immersion in 3% H_2_O_2_ peroxide for 25 min. Antigen unmasking was accomplished by incorporating slides for 1 h at 95°C in the target recovery solution. Tissue portions were blocked with 10% normal goat serum in phosphate-buffered saline after rapid cooling to room temperature. Antibodies for Nrf2 (#C20, Santa Cruz Biotechnology) were used for immunohistochemistry staining at dilution (1:2,000). 3,3-Diaminobenzidine (DAB) was used to develop and display colors. With hematoxylin, the tissue slices were gently counterstained, dehydrated, and covered. Using a light microscope, the slides were imaged.

To evaluate the production of macrophages in CA walls, the brain tissue in the area typically performed with CA was extracted and split into 5 μm sections. These areas were initially hydrated and then stained with primary antibody CD68 (CAS No. 3F103; 1:200 dilution, Santa Cruz Biotech, Shanghai, China), and consequently several secondary antibodies (CAS No. sc-2354; goat anti-mouse IgG, peroxidase-linked antibody, 1:5,000 dilution) were counterstained with hematoxylin. To ensure that a consistent number of macrophage cells were produced in the CA walls, the number of labeled positive cells was counted in a 100 μm square area surrounding the CA walls.

### 2.6 Statistical analysis

Mean ± SE was used to statistically measure the effects from multiple observations. Student’s *t*-test is used to deduce the significance of two mean values between two different groups. One-way ANOVA method was used for multiple comparisons. GraphPad Prism software was used to determine the significance with *P* < 0.05.

## 3 Results

### 3.1 PCA suppresses CA formation and progression in rats

In this study, we attempted to understand the inhibitory effect of PCA against CA progression, after the administration of elastase. The development of aneurysm was identified along the Willis circle or its major branches, which is consistent with previous studies [25,26,27]. Most aneurysms were larger in size, with multiple aneurysms around three to four times larger than their parent arteries. Before triggering CA, the experimental group of rats was treated with PCA. We found that the control group had an aneurysm size of 26.5 ± 0.76 μm, constantly increasing in size to 45.5 ± 1.67 μm (*P* < 0.001) in the group induced by intracranial aneurysm over a period of 16 weeks, whereas the group of rats pretreated with PCA had an aneurysm size significantly decreased to 31.33 ± 1.10 μm (*P* < 0.05) and 32.33 ± 2.06 μm (*P* < 0.01) at doses of 50 and 100 mg/kg, respectively, of PCA relative to the CA group (Table 2) in a dose-dependent manner. While taking into consideration the systolic blood pressure (SBP) levels, the CA group showed significant (*P* < 0.001) variation in their levels after 8 weeks of CA induction. Similarly, the group pretreated with PCA displayed a significant decrease in SBP levels after 8 weeks in a dose-dependent manner when compared to the CA group (Figure 1), besides the degree of elevated aneurysm scores (Table 3). Treatment with PCA suppressed vessel wall thickness in rats (*P* < 0.05) relative to the CA group (Table 4) in a dose-dependent manner. After CA induction, the body weight and BMI were substantially decreased after 4 weeks when compared to the control group. However, the groups receiving PCA-50 and 100 mg/kg treatments demonstrated a gain in body weight and BMI to normal control groups after 4 weeks. Furthermore, they retained the body weight and BMI of rats in groups receiving PCA treatments in a dose-dependent manner until 16 weeks of the study duration (Tables 5 and 6).

**Table 2:** Progression of CA size in control, induced, and PCA-50 and 100 mg/kg administered experimental group of rats monitored for 16 weeks

	Control	CA	PCA-50	PCA-100
0 week	28.33 ± 0.88	28.5 ± 0.76	27.5 ± 0.76	28.5 ± 0.76
4 weeks	26 ± 0.97	28.5 ± 0.76	29.5 ± 0.76	27.5 ± 0.76
8 weeks	26.5 ± 0.76	36.5 ± 0.76***	33 ± 0.97*	29.5 ± 0.76***
12 weeks	26.5 ± 0.76	38.5 ± 0.76***	31.33 ± 1.99**	30.67 ± 1.71**
16 weeks	26.5 ± 0.76	45.5 ± 1.67***	31.33 ± 1.10*	32.33 ± 2.06**

Values are expressed as mean ± SE (*n* = 16). Statistical significance is expressed as ***P < 0.001 CA compared to vehicle (control) and PCA-treated groups; *P < 0.05, PCA-50 compared to CA rats; and **P < 0.01 PCA-100 compared to CA rats.

**Figure 1:** Effect of PCA on systolic blood pressure in control, CA-induced, and experimental group of 16-week-monitored rats administered PCA-50 and 100 mg/kg. Values are expressed as mean ± SE (*n* = 16). Statistical significance is expressed as **P < 0.01; ***P < 0.01 compared to the control group, ^#^ *P* < 0.05 PCA-50 compared to CA rats, and ^Ψ^ *P* < 0.01 PCA-100 compared to CA rats.

**Table 3:** Effect of Nrf-2 activation on IA formation and progression with aneurysmal scores in control and PCA treatment groups

	CA	PCA-50	PCA-100
Aneurysmal score	3 ± 0.39	1.8 ± 0.21^*^	1.5 ± 0.2^**#^

Values are expressed as mean ± SE (*n* = 16). Statistical significance is expressed as *P < 0.05, PCA-50 compared to CA rats; **P < 0.01, PCA-100 compared to CA rats. ^#^ *P <* 0.05, PCA-100 compared with PCA-50 treatment. Aneurysmal scores in the CA group were much higher than that in the PCA group, corresponding to aneurysmal score of 1–5.

**Table 4:** Wall thickness ratio

	Control	CA	PCA-50	PCA-100
Wall thickness	38.5 ± 1.26	73.33 ± 1.71***	48.50 ± 4.0*	51.33 ± 2.81**

Values are expressed as mean ± SE (*n* = 16). Statistical significance is expressed as ***P < 0.001 CA compared to vehicle (control) and PCA-treated groups; *P < 0.05, PCA-50 compared to CA rats; and **P < 0.01 PCA-100 compared to CA rats.

**Table 5:** Effect of PCA-50 and 100 mg/kg administered to the experimental group of rats monitored for 16 weeks on body weight

	Control	CA	PCA-50	PCA-100
0 week	162.33 ± 2.45	165.5 ± 1.76	157.5 ± 2.36	158.5 ± 1.86
4 weeks	167.6 ± 1.97	138.5 ± 1.46**	159.5 ± 1.37*	157.5 ± 1.91*
8 weeks	163.5 ± 1.76	136.5 ± 2.46***	153.43 ± 1.97*	159.5 ± 2.76**
12 weeks	166.5 ± 1.36	135.5 ± 1.86***	161.33 ± 2.99**	168.67 ± 1.71***
16 weeks	167.5 ± 2.76	137.7 ± 2.67***	167.3 ± 1.10**	169.33 ± 2.06***

Values are expressed as mean ± SE (*n* = 16). Statistical significance is expressed as ***P < 0.001 CA compared to vehicle (control) and PCA-treated groups; *P < 0.05, PCA-50 compared to CA rats; and **P < 0.01 PCA-100 compared to CA rats.

**Table 6:** Effect of PCA-50 and 100 mg/kg administered experimental group of rats monitored for 16 weeks on BMI

	Control	CA	PCA-50	PCA-100
0 week	0.54 ± 0.005	0.55 ± 0.006	0.54 ± 0.003	0.54 ± 0.005
4 weeks	0.55 ± 0.007	0.50 ± 0.004**	0.54 ± 0.007**	0.54 ± 0.009**
8 weeks	0.54 ± 0.007	0.51 ± 2.46***	0.53 ± 0.009**	0.54 ± 0.006***
12 weeks	0.54 ± 0.003	0.50 ± 1.86**	0.54 ± 0.008**	0.55 ± 0.001***
16 weeks	0.55 ± 0.006	0.51 ± 0.006***	0.55 ± 0.002***	0.55 ± 0.006***

Values are expressed as mean ± SE (*n* = 16). Statistical significance is expressed as ***P < 0.001 CA compared to vehicle (control) and PCA-treated groups; *P < 0.05, PCA-50 compared to CA rats; and **P < 0.01 PCA-100 compared to CA rats.

The effect of PCA was examined in rats with H&E staining to assess the formation and progression of CA. A cerebral artery from the CA-induced group revealed that an endothelial cell lining with a thin layer of smooth muscle cells as described in Figure 2a and b shows moderately thick vascular walls with inflammatory infiltration of the cells, thus displaying distortion of the vessel wall with evidence of myointimal hyperplasia. The thickness of the tunica media in the PCA-treated groups was significantly decreased compared to the CA group (Figure 2c and d, Table 4) at 50 and 100 mg/kg in a dose-dependent manner.

**Figure 2:** H&E staining of normal cerebral artery, CA induced by elastase, and CA treated with PCA-50 and 100 mg/kg (a–h). Squares in f–h images are enlarged to show staining with anti-CD68-positive cells revealing that a majority of leukocytes in intracranial aneurysms were macrophages. 2G shows numerous leukocytes noticed in intracranial aneurysms indicating the distribution of macrophages was identical to that of leukocytes. Scale bar for a and e: 500 µm. Scale bar for b–d: 100 µm. Scale bar for f–h: 20 µm.

This study was able to analyze the effect of PCA on macrophage infiltration. Recruitment for macrophage infiltration was significantly (*P* < 0.05) elevated 4 weeks after aneurysm induction (Table 7, Figure 2f). Macrophage staining of the normal control group using anti-CD68 antibody in the cerebral artery showed lack of inflammatory cells and macrophage infiltration (Figure 2e). Chronic macrophage-related inflammation plays a major role in CA progression and can be seen in Figure 2f. This is further demonstrated with staining with anti-CD68 antibodies. The positive cells show that a majority of leukocytes in the intracranial aneurysms were macrophages. Figure 2f shows numerous leukocytes in intracranial aneurysms, and the distribution of macrophages was identical to that of leukocytes. Significantly, a fewer number of cells were observed at the inflammatory site as compared to CA after PCA treatments in a dose-dependent manner (*P* < 0.05) at 50 and 100 mg/kg, respectively (Table 7, Figure 2g and h).

**Table 7:** Macrophage infiltration (number of cells) in control, induced, and PCA-50 and 100 mg/kg administered experimental group of rats monitored for 16 weeks

	Control	CA	PCA-50	PCA-100
0 week	2.45 ± 0.12	2.26 ± 0.07	2.24 ± 0.06	2.35 ± 0.11
4 weeks	3.85 ± 0.09	4.09 ± 0.13	4.05 ± 0.13	4.05 ± 0.07
8 weeks	3.39 ± 0.08	7.02 ± 0.25***	5.57 ± 0.50*	5.37 ± 0.52**
12 weeks	4.78 ± 0.12	8.84 ± 0.19***	6.29 ± 0.68*	5.69 ± 0.81**
16 weeks	5.85 ± 0.12	8.92 ± 0.2***	6.93 ± 0.69*	6.41 ± 0.45**

Values are expressed as mean ± SE (*n* = 16). Statistical significance is expressed as ***P < 0.001 CA compared to vehicle (control) and PCA-treated groups; *P < 0.05, PCA-50 compared to CA rats; and **P < 0.01 PCA-100 compared to CA rats.

### 3.2 Effect of PCA on inflammatory cytokines, MMP-2, and MMP-9 analyzed by ELISA, qRT-PCR, and western blot analysis

The cytokine levels (Figure 3) in the group of rats induced with CA were elevated in comparison to the control group. The cytokines include IL-1β (*P* < 0.05), IL-2 (*P* < 0.05), IL-17 (*P* < 0.05), IL-8 (*P* < 0.01), IL-6 (*P* < 0.01), and TNF-α (*P* < 0.05). With the decline in the inflammatory cytokines in groups pretreated with PCA, the CA growth signaling was substantially (*P* < 0.05) reduced.

**Figure 3:** Effect of PCA on inflammatory cytokines in control, CA-induced, and experimental group of rats administered PCA-50 and 100 mg/kg. Values are expressed as mean ± SE (*n* = 16). Statistical significance is expressed as ***P < 0.01 compared to the control group, *P < 0.05 PCA-50 compared to CA rats, and **P < 0.01 PCA-100 compared to CA rats.

It’s been proved that the NF‑κB signaling was quite crucial in macrophage infiltration, and as a result, the levels of downstream MMP-2 and MMP-9 in the walls of aneurysm were measured. It was found that the levels of MMP-2 and MMP-9 proteins show an increase in the CA group and were reduced with PCA treatment (Figure 4).

**Figure 4:** Effect of PCA on relative expression of MMP-2 and MMP-9 in control, CA-induced, and experimental group of rats administered PCA-50 and 100 mg/kg. Values are expressed as mean ± SE (*n* = 16). Statistical significance is expressed as ***P < 0.001 compared to the control group, *P < 0.05 PCA-50 compared to CA rats, and **P < 0.01 PCA-100 compared to CA rats.

Growing evidence suggests that in chronic inflammation, there are molecular pathways causing TNF-α stimulation which further leads to nuclear translocation of NF-κB. This is also demonstrated in our studies where we found that NF-κB protein levels shown by western blot analysis (Figure 5) in aneurysmal walls of the CA were decreased in the rats treated with PCA-50 and 100 mg/kg. The data suggest that the TNF-α stimulated NF-κB pathway in macrophages was altered by PCA causing suppression of CA formation. Because of this, potentially, the NF‑κB pathway is involved in PCA to inhibit the progression of CA within macrophages (Figure 5).

**Figure 5:** Effect of PCA on relative mRNA expression of NF-κB in control, CA-induced, and experimental group of rats administered PCA-50 and 100 mg/kg. Values are expressed as mean ± SE (*n* = 16). Statistical significance is expressed as ***P < 0.01 compared to the control group, **P < 0.01 PCA-50 compared to CA rats, and ***P < 0.001 PCA-100 compared to CA rats.

To provide evidence of the protective role of PCA to CA, mRNA levels of transgelin (SM22) and inflammatory cytokines were analyzed with qPRC (Figures 3 and 6). The group of rats induced by the CA had elevated levels of cytokines TNF-α, IL-6, IFN-γ, and SM22. In contrast, a significant decrease in cytokine levels was observed in the PCA-treated groups (*P* < 0.01). Here, we validate the PCA’s protective action by inhibiting cytokines, thus proving it to be effective in controlling CA and therefore can be considered as a novel treatment (Figure 6).

**Figure 6:** Effect of PCA on inflammatory cytokines IFN-γ and SM22 in control, CA-induced, and experimental group of rats administered PCA-50 and 100 mg/kg. Values are expressed as mean ± SE (*n* = 16). Statistical significance is expressed as ***P < 0.01 compared to the control group, *P < 0.05 PCA-50 compared to CA rats, and **P < 0.01 PCA-100 compared to CA rats.

Nrf-2 pathway is involved in the mechanisms of antioxidant defense system. For the investigation of antioxidant enzymes such as NQO-1, qRT-PCR and western blot analysis were used. Figures 7 and 8 indicate that PCA increased the gene expression of antioxidant enzymes (Figure 8d–f), triggering Nrf-2 to substantially downregulate cytokine levels (*P* < 0.05) in both qRT-PCR and western blot analysis. Furthermore, our findings revealed that the activation of Nrf-2 with PCA in cytoplasm and nucleus as shown in Figure 7 shows a remarkable decrease in cytoplasmic Nrf-2 expression (Figure 8a and b) and an increase in nuclear Nrf-2 expressions (Figure 8a and c) after treatment with PCA, respectively (*P* < 0.05).

**Figure 7:** Effect of PCA on mRNA expressions of cytoplasm and nuclear fractions Nrf-2, antioxidant enzyme NQO-1 in control, CA-induced, and experimental group of rats administered PCA-50 and 100 mg/kg. Values are expressed as mean ± SE (*n* = 16). Statistical significance is expressed as ***P < 0.01 compared to control group, *P < 0.05 PCA-50 compared to CA rats, and **P < 0.01 PCA-100 compared to CA rats.

**Figure 8:** Effect of PCA on (a) and (d) western blot and (b, c, e, and f) densitometry analysis of cytoplasm and nuclear fractions Nrf-2 and antioxidant enzyme NQO-1 in control, CA-induced, and experimental group of rats administered PCA-50 and 100 mg/kg. Values are expressed as mean ± SE (*n* = 16). Statistical significance is expressed as ^#^ *P* < 0.01 compared to the control group, *P < 0.05 PCA-50 and 100 mg/kg compared to CA rats.

### 3.3 PCA causes downregulation and nuclear translocation of Nrf-2 with decreased cellular ROS levels

Nrf-2 expression was significantly decreased in the control group stained with DAB when compared to PCA treatment. There was a difference in expression between the cytoplasmic and nucleus cellular compartments in CA (Figure 9a). In the CA group, the amount of Nrf-2 found in the nucleus was greater than that of the group treated with PCA. Figure 9b shows that the CA group showed an increase in ROS levels visualized by an elevated fluorescence intensity (three-fold) when compared to the control group. This was substantially (*P* < 0.05) reduced by the treatment with PCA. These findings confirm that activation of Nrf-2 causes suppression of intracellular oxidative stress.

**Figure 9:** (a) Translocation of Nrf-2 from positive cells and number of positive cells analyzed (*n* = 4) showing H&E staining in CA-induced and PCA (100 mg/kg)-treated groups. (b) Intracellular ROS in the control, CA-induced, and experimental group of rats administered PCA-50 and 100 mg/kg. Values are expressed as mean ± SE (*n* = 16). Statistical significance is expressed as ***P < 0.01 compared to the control group, *P < 0.05 PCA-50 compared to CA rats, and **P < 0.01 PCA-100 compared to CA rats.

## 4 Discussion

This is the first study to investigate the effect of PCA on CA in rats. CA is a chronic inflammatory condition caused by excessive hemodynamic disturbance in arterial walls. It may cause serious SAH, a severe type of stroke. PCA possesses wide pharmacological activities such as anti-inflammatory, antioxidant, antiapoptotic, and anti-cancer [28,29,30,31]. Our findings demonstrated that PCA suppresses the formation and progression of CA via the inhibition of macrophage infiltration in rats when upon elastase administration. This mechanism has yet to be elucidated; however, several factors, namely hemodynamic stress, inflammation, degeneration of extracellular matrix, ROS generation, etc., contribute to the formation of CA [45]. In the CA group, elastic tissues with swollen aneurysmal dilation were absent. Furthermore, there was an increase in aneurysm size (Table 2) demonstrating the connection between the increase in size with the number of weeks after elastase administration. Our results showed that PCA treatment was able to reduce the effects of elastase significantly (P < 0.05) decreasing the aneurysm size, thereby showing the role of inflammatory cytokines, IL-1β, IL-2, IL-17, IL-8, IL-6 and TNF-α in the development of lesions in CA-induced rats (Figure 3) over 16 weeks.

Further validation of aneurysm induction using elastase was obtained by measuring systolic blood pressure in all animal groups. Our findings noted high blood pressure because of the induction of aneurysms over a period of 16 weeks. PCA treatment reduced the high blood pressure restoring readings comparable to control rats. The formation of CA was regulated by MMPs, namely MMP-2 and MMP-9, which caused the deterioration of the endothelium of cerebral arteries via degradation of elastic lamina resulting in inflammation and hypertension. The overexpression of MMP-2 and MMP-9 in CA-induced rats reinforced the effect of CA induction with elastase treatment relative to PCA groups. These overexpressions of MMPs that are involved in the progression of CA concur with results of other studies [46,47,48]. We investigated the role that the pro-inflammatory cytokine, TNF-α, plays in the development of intracranial aneurysm. The mRNA expression of pro-inflammatory cytokines, TNF-α, IL-17 IL-6, and IL-8 with activated infiltration of macrophages in response to IFN- γ, [49] showed a significant increase in CA-induced rats (Figure 6). The increase in IL-6 levels correlated with cerebral damage via the rupture of aneurysm and thus the development of CA [50]. Increased IL-1β levels in CA-induced rats demonstrated the deterioration of extracellular matrix, resulting in damage of the vascular endothelium [51]. The IL-1β levels were suppressed with PCA treatments and inhibited the development of an aneurysm, thus reducing the progression of vascular remodeling [52]. The recruitment of macrophage infiltration was demonstrated by an increase in IL-17 and IL-8 levels leading to the production of cytokines. These markers of inflammation result in the formation and development of aneurysm [53,54,55]. The increase in pro-inflammatory cytokines downregulated SM22, which in turn promoted the destruction and formation of the cytoskeleton and accelerated the formation and rupture of an aneurysm [56]. The treatment of PCA at 50 and 100 mg/kg showed a significant reduction in the levels of pro-inflammatory cytokines in a dose-dependent manner. This demonstrates that potentially TNF-α signaling mechanism is involved in the development and progression of CA.

In addition, PCA was shown to inhibit NF-κB expression, subsequently exerting anti-inflammatory action on aneurysms. Our results show an increase in systolic pressure denoting induction of hemodynamic stress in animal models within the intracranial arteries, thereby triggering inflammation with progression of CA, similar to the pathogenesis of CA in humans [57].

Although several studies reported the role of NF-κB as a key transcription factor in the regulation of the expression of MMPs, production and release of pro-inflammatory cytokines, and macrophage infiltration in advancing the progression of CA [58,59,60], the effect of PCA on the CA progression has not been reported. The treatment with PCA at the two different doses shows suppression in aneurysmal wall degeneration, prevention in macrophage infiltration, and inflammatory cytokines. This potentially involves the role of NF-κB and MCP‑1 signaling pathways and could be a therapeutic target in the treatment of CA. In addition, this study noticed significant reductions in the expressions of MMP-2 and MMP-9 in PCA-treated groups. While CA pathogenesis involving MMPs is debated, our findings concur with a previous study, showing an increased expression of MMP-2 and MMP-9 in human serum and aneurysmal walls [61].

Inflammation and oxidative stress are possibly involved in causing endothelial dysfunction. The transcription factor, Nrf-2, is involved in the modulation of cellular oxidative processes via antioxidant and detoxifying genes. Under oxidative stress, Nrf-2 translocates from the cytoplasm to the nucleus. Thus, we hypothesized that the potential role of Nrf-2 activation is to inhibit the oxidative stress and offer protective effects against CA formation and progression. Our results showed reduced aneurysmal scores and progression of CA without rupturing after treatment with PCA at 50 and 100 mg/kg, respectively, thus indicating the role of Nrf-2 pathway activation in the suppression of CA progression. This is consistent with another study that reported elevated Nrf-2 levels in the inhibition of acute aortic dissection formation. Our immunohistochemical findings showed the downregulation and Nrf-2 nuclear translocation in aneurysm walls (Figure 9).

We show that PCA decreases the inflammatory responses in the formation of CA by inhibiting the NF‑κB pathway and macrophage infiltration. NF‑κB pathway inhibition can be a potential target for the prevention and treatment of CA. We also confirmed that Nrf-2 signaling inhibits CA formation and development, via acting on Nrf-2 translocation into the nucleus. TNF-α signaling initiates the procedure in the CA-induced group of rats by development and maturation of the CA. We found that with the treatment of PCA, it is possible to control aneurysms as well as inhibit the aneurysm rupture in the brain (Figure 10).

**Figure 10:** Schematic representation of the study.

## 5 Conclusion

This study suggests that formation and progression of CA induced by inflammation and oxidative stress can be inhibited with the treatment of PCA in a dose-dependent manner. This involves the regulatory roles of TNF-α, NF-κB, and Nrf-2 activation pathways. The underlying mechanism involves a decreased expression of pro-inflammatory cytokines, upregulation of antioxidant enzyme activities, and reduced intracellular ROS formation. We propose that PCA can be an alternative and novel therapeutic for the treatment of CA by inhibiting TNF-α, NF-κB, and Nrf-2 activation pathways.
